The article "Short course hypofractionated whole breast irradiation after conservative surgery: a single institution phase II study" was published in 2017. Journal: J Exp Clin Cancer Res.

# Short course hypofractionated whole breast irradiation after conservative surgery: a single institution phase II study

**DOI:** 10.1186/s13046-017-0640-z

**Published:** 2017-12-27

**Authors:** Paola Pinnarò, Carolina Giordano, Alessia Farneti, Adriana Faiella, Giuseppe Iaccarino, Valeria Landoni, Diana Giannarelli, Patrizia Vici, Lidia Strigari, Giuseppe Sanguineti

**Affiliations:** 1 Departments of Radiation Oncology, Regina Elena National Cancer Institute, Via Elio Chianesi 53, 00144 Rome, Italy; 2 Laboratory of Medical Physics and Expert Systems, Regina Elena National Cancer Institute, Rome, Italy; 3 Departments of Statistics, Regina Elena National Cancer Institute, Rome, Italy; 4 Departments of Clinical Oncology, Regina Elena National Cancer Institute, Rome, Italy

**Keywords:** Breast neoplasms, Breast carcinoma in situ, Radiotherapy, Dose hypofractionation, Local neoplasm recurrence

## Abstract

**Background:**

To assess the oncologic outcomes of hypofractionated whole breast irradiation (Hypo-WBI).

**Methods:**

Eligible patients had undergone breast conservative surgery for early breast cancer (pTis-2) and none/limited nodal involvement. Hypo-WBI consisted of 34 Gy in 10 daily fractions over 2 weeks to the whole breast three-dimensional conformal radiotherapy (3DCRT), followed by a single fraction of 8 Gy to the tumor bed after 1 week (electrons). Primary endpoint is freedom from ipsilateral breast tumor recurrence (IBTR). Minimum follow up for living & event-free patients is 3 yrs.; median follow up time of the whole analyzed patient population is 5.4 yrs. (range: 1.8–11.4 yrs).

**Results:**

Two hundred fifty-one patients were accrued from 2004 to 2013. All patients underwent local excision of the primary tumor to negative margins. Four patients failed in the ipsilateral breast after a median time of 3.2 years (range: 1.7–5.7 yrs) for a 5-year IBTR-free survival of 98.7% (95%CI: 97.3%–100%). IBTR-free survival was significantly higher for patients with invasive cancer than for patients with intraductal carcinoma (*p* = 0.036). Within patients with invasive tumors, no clear trends or associations were detected between IBTR and age, grading, molecular subtype, pT or pN stage. At 5 years, the actuarial rates of GR2 fibrosis and GR2+ teleangectasia are 2.4% (95%CI: 0–6.5%) and 7.1% (95%CI: 0.4–13.7%), respectively. Cosmesis was scored as excellent/good by ≈95% of patients and ≈60% of clinicians.

**Conclusions:**

Hypo-WBI in 3 weeks allows excellent oncologic outcomes for invasive breast cancer after conservative surgery. Patients with intraductal carcinoma should be treated with Hypo-WBI only within a controlled study.

**Trial registration:**

IRE-IFO Ethical and Scientific Committee (cod. RS61/04).

The article "Short course hypofractionated whole breast irradiation after conservative surgery: a single institution phase II study" was published in 2017. Journal: J Exp Clin Cancer Res.

## Background

Breast cancer is the most commonly diagnosed malignancy in females in the US, with almost 250,000 women diagnosed per year [1]. A large proportion of patients presents with early-stage disease and is candidate for breast-conserving therapy. Postoperative whole-breast irradiation (WBI) is the standard of care for these patients [2]. Conventionally fractionated regimens traditionally deliver WBI over approximately 5 weeks in 25–28 fractions to doses of 45–50 Gy. Further improvements in local control rates can be achieved for many patients with additional dose of radiation to a limited volume of the breast (“boost”) [3] extending the treatment course by approximately 1 to 2 weeks to an overall treatment time of 6 to 7 weeks. Instead of following WBI completion, the boost can be delivered at each fraction as ‘simultaneous integrated boost’ [4] thus avoiding further treatment extension beyond WBI.

In attempt to improve efficiency, cost of care delivery as well as patient logistics, alternate techniques and dose scheduling have been investigated. Randomized clinical trials in Canada and the UK have demonstrated that shorter treatment regimens (3 to 4 weeks) may be as safe and effective as conventional schedules [5–7]. However, there has not been significant adoption of hypofractionated WBI (Hypo-WBI) in the United States [8]. Since the above trials have selected low-risk patients, one concern is whether Hypo-WBI can be offered to patients at higher risk of in-breast failure [4]. Other concerns potentially limiting the use of Hypo-WBI are the use of a boost and its timing relative to WBI [4]. None of the prospective trials for Hypo-WBI systematically delivered a tumor bed boost; in the START A and B trials it was left to the Institutional policy, so it was delivered in only a fraction of patients and in a nonrandomized fashion. Moreover, the use of a sequential boost of 1–2 weeks after WBI extends the overall treatment time reducing the potential time-saving benefit from hypofractionation.

In 2004 we designed a novel treatment schedule of Hypo-WBI in which therapy was completed in 11 fractions over 3 weeks inclusive of a sequential single-fraction boost. After a preliminary phase I part [9], in the present study we report the outcomes of 251 patients at a minimum follow up of 3 years.

## Methods

### Study description

This is a prospective phase II study evaluating the efficacy of a novel Hypo-WBI schedule. Inclusion criteria were: age > 18 years; pathologically proven breast carcinoma undergone complete local excision within a breast conserving strategy to negative margins (R0); pathological primary tumor stage up to pT2 (pTis-pT2); pathological nodal stage up to pN1a (pNx-pN1a); no distant metastases (M0); no previous local surgical or radiation treatment; no previous chemotherapy; specific informed consent. The study was approved by the local Institutional Ethical and Scientific Committee (cod. RS61/04). All patients provided a written informed consent.

The article "Short course hypofractionated whole breast irradiation after conservative surgery: a single institution phase II study" was published in 2017. Journal: J Exp Clin Cancer Res.

The study opened to accrual in October 2004 and was initially offered only to selected patients unable to undergo conventional adjuvant radiotherapy in 6–6.5 weeks due to logistic reasons or refusal [9]. This pilot phase lasted until March 2006, when 39 patients had been accrued [9]. After preliminary toxicity data showed its feasibility, this schedule has been offered to all patients operated conservatively for early breast cancer at our Institution and satisfying the above criteria since June 2008.

### Immunohistochemistry data

Histologic grade was scored according to the Nottingham system. Estrogen receptor (ER) status, progesterone receptor (PR) status and proliferation rate (ki67) were assessed throughout immunohistochemistry (IHC). Human epidermal growth factor receptor 2 (HER2) status was initially assessed with IHC. Tumors were considered HER2+ if they received a score of 3+ on IHC staining or if they received a score of 2+ by IHC staining and showed HER2 amplification based on silver-enhanced in situ hybridization (SISH) [10]. Tumors with scores of 2+ by IHC staining in the absence of SISH amplification were considered HER2 negative.

Patients were categorized based on the receptor status of their primary tumor: luminal A (ER+ or PR+ and HER2- and ki67 < 20%), luminal B (ER+ or PR+ and HER2+ or ki67 ≥ 20%), HER2-enriched (ER- and PR- and HER2+), and triple negative/basal (ER- and PR- and HER2-).

### Radiotherapy technique

The details of radiotherapy technique have been reported previously [9]. Briefly, Hypo-WBI consisted of 34 Gy in 10 daily fractions over 2 weeks to the whole breast, followed by a single fraction of 8 Gy. When the schedule was designed no information was available on the (acute) tolerance to Hypo-WBI. Therefore, one-week gap between the end of Whole Breast irradiation and the boost was planned in order to allow the recovery of normal breast tissues from Hypo-WBI. Despite the preliminary excellent results in terms of acute toxicity [9], the gap was maintained for logistic reasons and it became part of our institutional practice. The regional lymph nodes were not intentionally targeted. Whole breast parenchyma was covered by two tangential fields, 6 MV photon beams 3D–CRT. Wedge compensation was used to ensure a uniform dose distribution to the target volume within −5% and +7%. Moreover, 95% of the prescribed dose had to be received by at least 95% (goal) of the planning target volume (PTV), or by 90% of the PTV as acceptable variation; while maintaining a maximum lung depth ≤ 2.5 cm.

The article "Short course hypofractionated whole breast irradiation after conservative surgery: a single institution phase II study" was published in 2017. Journal: J Exp Clin Cancer Res.

The boost dose of 8 Gy (prescribed to the 90% reference isodose) was administered via a 6 to 12 MeV appositional electron field.

### Study endpoints

The primary endpoint of the present study is freedom from ipsilateral breast tumor recurrence (IBTR). Local tumor relapse was defined as any breast quadrant local relapse. Any ipsilateral regional relapse outside the radiotherapy target volume was excluded from the analysis of local relapse.

This study was designed to assess the 5-year IBTR rate. On the basis of available literature at the time of the design of the study we assumed a 5% rate [3]; a sample size of 250 patients would have been able to estimate this percentage with a standard error of 1.38%.

Secondary endpoints include freedom from contralateral breast tumor recurrence (CBTR), from distant metastases (DM) and from second (non-breast) primary tumors. Progression free survival includes any of the above events as well as death due to inter-current causes.

Late toxicity was scored according to the LENT/SOMA [11] and CTCAE v4.0 [12] scales as appropriate. The highest level of reaction in any quadrant of the treated breast was considered the final grade. Toxicity grades could be pooled and dichotomized in order to perform further analysis as detailed below. Cosmesis was scored independently by two observers according to the Harvard scale after reviewing the pictures at the last follow up [13].

### Statistical analysis

Distributions of covariates between samples were analyzed by contingency tables (chi square test) and by non-parametric tests (Mann U Whitney). Actuarial curves are computed with the Kaplan-Meier method from the last day of radiotherapy. Patients were still evaluable for local-regional relapse after distant relapse, but were censored at date of death. Estimates of 5-year events were calculated (with 95% Confidence Intervals-CIs). The log-rank test was used to compare survival distributions. Cox proportional hazard regression model was used to estimate hazard ratios (HR) and their 95% confidence intervals. Within the subgroup of invasive tumors, selected covariates were investigated at univariate analysis for a possible association with the time to IBTR: age (continuum); grading (G3 vs others); primary tumor stage (pT1 vs pT2); nodal stage (pN0 vs pN1a); molecular profile (Luminal vs Her2 enriched vs Triple negative). Significance was claimed for *p* values below 0.05. Estimation of the 95% confidence intervals for proportions was done with the Wilson score method. Inter-rater agreement for was estimated through the Cohen’s kappa (κ). The κ value indicates no (κ = 0), slight (κ = 0–0.2), fair (κ = 0.2–0.4), moderate (κ = 0.4–0.6), substantial (κ = 0.6–0.8) or almost perfect (κ = 0.8–1) agreement.

The article "Short course hypofractionated whole breast irradiation after conservative surgery: a single institution phase II study" was published in 2017. Journal: J Exp Clin Cancer Res.

Minimum follow up for living & event-free patients is 3 yrs.; median follow up time of the whole analyzed patient population is 5.4 yrs. (range: 1.8–11.4 yrs).

## Results

### Patients & treatment

From October 2004 to August 2013, 251 patients were accrued. Selected patient, tumor and treatment characteristics are reported in Table 1. Mean age is 61.1 yrs. (SD: 12.2). Overall, 52 (20.7%), 58 (23.1%), 67 (26.7%) and 44 (17.5%) patients were younger than 50 years, had pT2 primary tumors, had poorly differentiated tumors (G3), were nodal positive (pN1a), respectively. Slightly more than 10% of patients had in-situ ductal carcinoma (pTis). Of them, 13 (46.8%) received also adjuvant hormonal treatment. All patients underwent local excision of the primary tumor to negative margins. Twenty patients did not undergo surgical staging of the axilla (pNx), including 16 patients with DCIS, 1 patient with pT1mic, 2 patients with pT1c and 1 patient with pT2 disease. All patients with pN1a disease underwent dissection of at least levels I and II of the ipsilateral axilla.

**Table 1:** Selected characteristics of the patients, tumors and treatments

Covariate	Stratification	N	%
Tumor Location	Superior Half	189	75.3
	Inferior Half	62	24.7
Pathology	DCIS	28	11.2
	Ductal	202	80.5
	Lobular	10	4.0
	Mixed	5	2.0
	Other	6	2.4
Grading	G1	34	13.5
	G2	136	54.2
	G3	67	26.7
	Gx	14	5.6
Estrogen Receptors	Negative	39	15.5
	Positive	210	83.7
	Unknown	2	0.8
Progesterone Receptors	Negative	59	23.5
	Positive	190	75.7
	Unknown	2	0.8
Menopausal Status	Premenopausal	70	27.9
	Postmenopausal	181	72.1
Axilla staging	SNB(OSNA method [33, 34])	143	57.0
	AND	88	35.0
	None	20	8.0
pT Stage	DCIS	28	11.2
	pT1mic	4	1.6
	pT1a	15	6.0
	pT1b	37	14.7
	pT1c	109	43.4
	pT2	58	23.1
pN Stage	pN0	180	71.7
	pNmic	7	2.8
	pN1a	44	17.5
	pNx	20	8.0
Adjuvant tmt	None	20	8.0
	Hormones	132	52.6
	Chemotherapy	31	12.4
	Chemotherapy + Hormones	68	27.1

Abbreviations: *SNB* sentinal nodal biopsy, *OSNA* one step nucleic acid amplification, *AND* axillary nodal dissection, *DCIS* Ductal carcinoma in situ, *pT* Primary tumor stage at pathology, *pN* Nodal stage at pathology, *tmt* treatment

Molecular profile was assessed in the 223 patients with infiltrative lesions (Table 2). Of the 41 patients with HER2 positive status, 31 (75.6%) received Herceptin as part of their adjuvant systemic treatment. Overall, of 99 patients undergoing adjuvant chemotherapy, most patients (86.8%) received anthracycline- and/or taxane-based chemotherapy. None of the patients underwent neoadjuvant chemotherapy.

The article "Short course hypofractionated whole breast irradiation after conservative surgery: a single institution phase II study" was published in 2017. Journal: J Exp Clin Cancer Res.

**Table 2:** Molecular profiling of patients with invasive breast cancer (*N* = 223)

Covariate	Stratification	N	%
Ki-67	<20%	141	63.2
	≥20%	81	36.3
	Unknown	1	0.4
HER2 status	Negative	182	81.6
	Positive	41	18.4
Molecular groups	Luminal A	127	57.0
	Luminal B	59	26.5
	HER2 enriched	17	7.6
	Triple Negative	19	8.5
	Unclassified	1	0.4

Abbreviations: *HER2* Human epidermal growth factor receptor 2

All patients completed the planned radiation treatment including the boost. Mean treatment duration (including the boost) was 2.9 weeks (95%CI: 2.5–3.3 weeks). The median PTV volume of the breast was 549 cm^3^ (range 113–2118 cm^3^). WBI treatment plans were normalized to intentionally keep the maximum dose below 107% of the prescribed dose. Nevertheless the median volume receiving a total dose higher than 107% (V36.4Gy) of the prescription dose (34 Gy) was less than 0.01 cm^3^ (range: 0.0–5.3 cm^3^). Therefore, the median prescribed dose was 33.8 Gy (range: 32.5–34.4 Gy). The median mean lung dose was 2.7 Gy (range: 0.5–6.4 Gy). For left-sided tumors, the median mean heart dose was 0.8 Gy (range: 0.2–3.6 Gy) and the median heart V3 Gy was 7.3 cm^3^ (range: 0.0–148.5 cm^3^).

### Oncologic outcomes

Four patients developed a local failure after a median time of 38.4 months. Estimated 5-yr. IBTR-free survival is 98.7% (95%CI: 97.3–100%) (Fig. 1). All observed local failures were infiltrative and in the original quadrant. Selected characteristics of the patients developing a local failure are reported in Table 3.

**Fig. 1:** IBTR-free survival for the overall population

**Table 3:** Selected patient, tumor and treatment characteristics for patients who developed a IBTR

Initials	Age (years)	Grade	Path	pT	pN	ER/PR status	Ki-67	HER2 status	Molecular Group	Systemic tmt	Time to IBTR (months)
F.R.	45	3	D	is	X	NA	NA	NA	NA	None	68.8
A.A.	68	3	D	is	0	Positive	NA	NA	NA	None	45.9
R.B.	50	2	D	2	1a	Positive	5%	Negative	Luminal A	Chemo-horm	30.6
D.M.	56	2	D	2	0	Positive	40%	Positive	Luminal B	Chemo-horm	20.2

Abbreviations: *IBTR* ipsilateral breast tumor recurrence, *HER2* Human epidermal growth factor receptor 2, *pT* Primary tumor stage at pathology, *pN* Nodal stage at pathology, *tmt* treatment, *D* invasive ductal carcinoma

IBTR-free survival was significantly higher for patients with invasive cancer at diagnosis than for patients with intraductal carcinoma (5-yr. IBTR-free survival 99.1%, 95% CI: 97.9–100% and 95.2%, 95%CI: 86.2–100%, respectively, *p* = 0.036, Fig. 2).

**Fig. 2:** IBTR-free survival for invasive and ductal carcinoma in situ (DCIS). Considering the DCIS subgroup as the reference one, the Hazard Ratio (HR) of IBTR for the invasive group is shown

Within invasive tumors, no clear trends or associations were detected between the time to IBTR and age (continuum) (*p* = 0.362), grading (*p* = 0.617), primary tumor stage at pathology (pT2 vs pT1)(*p* = 0.471) or lymph node stage at pathology (pN0 vs pN1a)(*p* = 0.89) and molecular profile (Triple negative vs HER-2 enriched vs Luminal A-B)(*p* = 0.70).

The article "Short course hypofractionated whole breast irradiation after conservative surgery: a single institution phase II study" was published in 2017. Journal: J Exp Clin Cancer Res.

Four patients developed distant metastases and, of them, 2 died of disease. Five-year DM-free survival is 98.1% (95%CI: 97.9–98.3%). Five patients developed a contralateral breast cancer, 4 infiltrative and 1 ductal carcinoma in situ after a median time of 45.6 months (range: 9.6–80.4 months). Five-year CBRT-free survival is 98.7% (95%CI: 97.3–100%). Thirteen patients developed a second primary tumor (which was lethal in 3) and 3 additional patients died of intercurrent disease. Five-year overall and progression free survivals are 96.7% (95%CI: 94.2–99.2%) and 91.6% (95%CI: 87.9–95.3%), respectively.

### Toxicity & Cosmesis

Five patients developed peak grade 2 fibrosis (CTCAE v4.0) of the treated breast. Eighteen patients developed skin teleangectasia (LENT/SOMA): grade (GR) 2 and GR3 in 11 and 7 patients respectively. Figure 3 shows the time to GR2 fibrosis and GR2+ teleangectasia, respectively. At 5 years, the actuarial rates of GR2 fibrosis and GR2+ teleangectasia are 2.4% (95%CI: 0–6.5%) and 7.1% (95%CI: 0.4–13.7%), respectively. No other GR2+ reaction has been recorded.

**Fig. 3:** Cumulative rates of both GR2 fibrosis and GR2+ teleangectasia

Cosmesis was assessed at a mean (SD) time of 63.7 (26.5) months after treatment end on 223 (88.8%) of patients. Results are illustrated in Fig. 4. Regarding physician-reported scores, slightly more than 60% of patients were judged to have an excellent or good cosmetic appearance by either observer. Conversely, ≈15% of patients were considered to have a poor cosmetic outcome. The inter-observer agreement is substantial (κ = 0.648, *p* < 0.001). According to patient-reported scores, the majority of patients (94.2%) felt to have an excellent or good cosmetic outcome. There was no correlation between patient and physician scores (κ = −0.007 and κ = 0.022 between patients and observer 1 and between patients and observer 2, respectively).

**Fig. 4:** Cosmetic outcomes according to both clinicians (obs 1 and obs2: observer 1 & 2) and patients (PRO: patient reported outcomes)

## Discussion

The results of the present prospective single-Institution study confirm Hypo-WBI to be an effective option after breast conserving surgery for early stage invasive breast carcinoma. Our 5-year estimate of IBTR is comparable to the ones obtained within selected phase III studies at a similar length of follow up (Fig. 5). Local recurrence is usually higher between years 3 and 5 of follow up, with 2/3 of local failures taking place within 5 yrs. [14]. Therefore, even if further IBTR events are to be expected, we believe that our results are reasonably mature with regard to this endpoint.

The article "Short course hypofractionated whole breast irradiation after conservative surgery: a single institution phase II study" was published in 2017. Journal: J Exp Clin Cancer Res.

**Fig. 5:** Five-yr. IBTR (95%CI) from randomized controlled studies along with the present study (Invasive ca only)(IRE: Regina Elena Institute). The experimental arms of each study were as follow: OCOG (Ontario Clinical Oncology Group Trial), 42 Gy/16 fractions/3.2 wks, median follow up 5.75 yrs., 622 pts. [5]; START P (Standardization of Radiotherapy Pilot) trial, 39 Gy/13 fractions/5 wks and 42.9 Gy/13 fractions/5 wks, median follow up 9.7 yrs., 474 and 466 patients, respectively [12]; START A trial, 39 Gy/13 fractions/5 wks and 41.6 Gy/13 fractions/5 wks, median follow up 5.1 yrs., 737 and 750 patients, respectively [4]; START B trial, 40 Gy/15 fractions/3 wks, median follow up 6.0 yrs., 1110 patients [3]

The Cox proportional hazard regression of both START-P and START-A trials allowed a direct estimate of the radiosensitivity (α/β ratio) for tumor local recurrence at 3.5 Gy (95%CI: 1.3–5.7 Gy) [15]. When applied to the present schedule, 34 Gy in 10 fractions would be equivalent to 42.6 Gy (95%CI: 40.2–48.4 Gy) delivered at 2.0 Gy fractions (EQD2 Gy), assuming no impact of treatment time. In other words, disregarding the effect of shortening the treatment time from 5 to 2 weeks, 34 Gy in 10 fractions would correspond to 42.6 Gy in 21.3 fractions. When the treatment time is factored in by considering a daily dose of 0.60 Gy necessary to compensate for each saved day of treatment (Dprolif = 0.60 Gy/day, 95%CI: 0.10 to 1.18 Gy/day) [16], the EQD2 Gy for WBI jumps to 55.2 Gy (95%CI: 50.5–65 Gy). Interestingly, despite similar (but not identical) entry criteria, Fig. 5 shows that the most favorable IBTR rates have been achieved within studies investigating schedules that shorten WBI by 2–3 weeks such as the IRE, OCOG and START B ones.

The role of a boost dose to the tumor bed in the setting of hypofractionated WBI remains unclear. In 2011, the ASTRO task force recommended not to use hypofractionated RT when a tumor bed boost was thought to be indicated due to the lack of data at that time [17]. In the earlier part of START-P trial, there was a sub-randomization between boost (14 Gy in 7 fractions, 364 pts) and no boost (359 pts) after WBI. Unfortunately, no clinical results have been disclosed [14]. In the following START trials the use of a boost (10 Gy/5 fractions) after WBI was left to each Institution policy and, overall, ≈50% of patients received it. Conversely, in the OCOG trial, excellent IBTR rates have been achieved without a boost [7].

The article "Short course hypofractionated whole breast irradiation after conservative surgery: a single institution phase II study" was published in 2017. Journal: J Exp Clin Cancer Res.

In our experience a tumor bed boost was always delivered regardless clinical/tumor factors and thus it became integral part of the treatment schedule. By applying the same parameters as above, 8 Gy in single fraction corresponds to an EQD2 Gy of 9.2 Gy (95% CI: 7.4–11.0 Gy) for a cumulative tumor bed dose in 3 weeks of 61.1 Gy (95%CI: 44.8–77.4 Gy). In other words, it is estimated that, on average, the tumor bed boost adds only 5 more Gy at 2 Gy due to the week break after WBI. Since the slope of the dose–response at the IBTR rates observed here is very shallow [16], we doubt that such a limited increase in the total dose had a large effect on local control. Therefore, one option would be to discontinue the systematic use of the boost, reserving it only for selected patients (i.e. those with high grade tumors and those with an intraductal component). Moreover, in this case, in order to maintain a reasonably high biological effective dose, it might be worth to consider delivering the boost right after WBI (avoiding any break) or to investigate a concurrent boost delivery technique (‘simultaneous integrated boost’) as others have successfully explored [4].

Multiple studies have suggested that the molecular tumor profile predicts for IBTR after conventional RT [18, 19]. However, there are limited data on the efficacy of hypofractionation by breast cancer molecular subtype [20]. Post-hoc analysis on 989 patients (80%) accrued within the OCOG study for whom formalin-fixed paraffin-embedded tumor block were available, showed that molecular subtype was the only predictor of local recurrence at multivariable analysis. The 10-yr. IBTR rates were 4.5% for luminal A and basal-like, 7.9% for luminal B and 16.9% for HER2 enriched tumors (*p* < 0.01) [20]. Moreover, no evidence of an interaction between RT fractionation (hypofractionated or standard) and molecular subtype was observed for IBTR [18]. Contrary to the OCOG and other studies [18, 19], in the present one trastuzumab was considered for patients with HER2 tumors, and this may have compensated for the poorer prognosis of HER2 enriched tumors [21]. A longer follow up on a larger number of patients is needed to confirm this finding.

A recent meta-analysis tried to clarify the role of hypofractionation for ductal carcinoma in situ (DCIS) [22]. Since DCIS tumors were not included in any prospective randomized study on hypofractionation, the Authors analyzed 4 observational studies comparing IBTR rates between patients who received standard vs hypofractionated RT (2534 pts) finding no difference in local recurrence rate by fractionation despite a trend in favor of hypofractionation (OR: 0.78, 95% CI: 0.58–1.03, *p* = 0.08) [22]. An ongoing phase III study (NCT00470236) by the Trans-Tasman Radiation Oncology Group is trying to clarify the issue. In the meantime, the present data raise caution when treating patients affected by DCIS with hypofractionation.

The article "Short course hypofractionated whole breast irradiation after conservative surgery: a single institution phase II study" was published in 2017. Journal: J Exp Clin Cancer Res.

Teleangectasia and fibrosis are the most prevalent late side effects after breast irradiation [23]. Fibrosis incidence is maximal during the first few years after treatment and then plateaus [24] while skin teleangectasia shows a progressive onset at least up to 10 yrs. after treatment [25]. Therefore, the rate of mild fibrosis observed in the present study (2.4% with an upper 95% limit of 6.5%) along with the lack of severe (GR3) toxicity seems particularly favorable and similar if not better than historical controls at comparable time-points [26]. Since the risk of fibrosis seems related to the maximal dose delivered during whole breast irradiation rather than volume parameters [24], we believe that the fact that our WBI treatment plans were highly homogeneous may have had a major role in reducing its occurrence.

It has been shown that, for a given fractionation schedule, fibrosis and telangiectasia develop independently within the same patient [27] and have different predictors [28, 29]. Accordingly, the estimated 5-yr. rate of GR2+ teleangectasia (7.1%, upper 95% limit: 13.7%) was higher than GR2 fibrosis (Fig. 3), though it seems comparable to the rate (12.4%) reported in the boost arm of the Lyon trial at the same time point [28]. We have previously shown that selected boost parameters (area and electron energy) are independently correlated to the risk of GR2+ telangiectasia [9]. Therefore, it is possible that changing boost strategy (both indication and technique, as previously discussed) will reduce the prevalence of GR2+ teleangectasia.

Similar to other studies [30, 31], the overall concordance between clinicians and patients in scoring toxicity was low. Moreover, we found that, on average, patient perception of toxicity is more optimistic than physician one. Overall, the vast majority of patients felt to have had an excellent or good cosmetic outcome, while the rate dropped to ≈60% when scored by the physician. Though using different scales, others have reported similar rates for physician reported outcomes. In the OCOG study, cosmetic outcome according to the EORTC Cosmetic rating System on 448 patients treated within the short arm was excellent or good in 77.9% of patients at 5 years [7]. In the START P trial at a minimum follow up of 5 years, physician-scored excellent/good cosmetic results were reported in 54.6% and 37.9% of patients after 39 Gy and 42.6 Gy, respectively [32].

The article "Short course hypofractionated whole breast irradiation after conservative surgery: a single institution phase II study" was published in 2017. Journal: J Exp Clin Cancer Res.

## Conclusion

In conclusion, the results of this single-Institution prospective study on 251 patients at a minimum follow up of 3 yrs. show that Hypo-WBI is associated with a very low risk of both IBTR and long term toxicity as well as with good to excellent cosmetic outcomes in most of the patients. Though both oncologic and morbidity outcomes will be continuously monitored, 34 Gy in 10 fractions to the whole breast followed by a single dose boost are currently offered as standard treatment at our Institution for all the patients with invasive cancer after breast conservation surgery who fit the above inclusion criteria. The present results also suggest that the delayed single-fraction boost may be safely omitted, and this in turn may reduce the risk of skin teleangectasia, though this deserves prospective confirmation among properly selected (low risk) patients. Finally, for patients with DCIS, the present data do not support treatment with Hypo-WBI outside a controlled/research study.

## Abbreviations

3D–CRT: Three-dimensional-conformal Radiotherapy
AND: Axillary nodal dissection
CBTR: Contralateral breast tumor recurrence
D: Invasive ductal carcinoma
DCIS: Ductal carcinoma in situ
DM: Distant metastases
EQD2 Gy: Equivalent dose delivered at 2.0 Gy fractions
ER: Estrogen receptor
HER2: Human epidermal growth factor receptor 2
Hypo-WBI: Hypofractionated WBI
IBTR: Ipsilateral breast tumor recurrence
IHC: Immunohistochemistry
ki67: Proliferation rate
OSNA: One step nucleic acid amplification
pN: Nodal stage at pathology
PR: Progesterone receptor
pT: Primary tumor stage at pathology
SD: Standard deviation
SISH: Silver-enhanced in situ hybridization
SNB: Sentinal nodal biopsy
tmt: Treatment
WBI: Whole-breast irradiation
